This article has been retracted.

# IGF-1 Promotes Epithelial-Mesenchymal Transition of Lens Epithelial Cells That Is Conferred by miR-3666 Loss

**DOI:** 10.1155/2022/5383146

**Published:** 2022-07-14

**Authors:** Chao Wang, Baowen Zhao, Jiahui Fang, Zhan Shi

**Affiliations:** ^1^The First Affiliated Hospital of Harbin Medical University, Anesthesiolgy Department, Harbin, China; ^2^Hongqi Hospital Affiliated to Mudanjiang Medical College, Ophthalmology Department, Mudanjiang, China; ^3^The First Affiliated Hospital of Harbin Medical University, Ophthalmology Department, Harbin, China

## Abstract

The abnormal proliferation, migration, and epithelial-mesenchymal transformation (EMT) of lens epithelial cells (LECs) are the main reasons for vision loss caused by posterior capsular opacification (PCO) after cataract surgery. Insulin-like growth factor-1 (IGF-1) was found to be associated with the pathogenesis of cataracts, but its biological role in PCO is poorly understood. In the present study, IGF-1 overexpression facilitated the proliferation, migration, and EMT, whereas knockdown of IGF-1 markedly suppressed the proliferation, migration, and TGF-*β*2-induced EMT of LECs. Additionally, to evaluate valuable microRNAs (miRNAs) which target IGF-1 to modulate LEC-EMT, we predicted miR-3666 might regulate IGF-1 by binding its 3'UTR according to the bioinformatics database. Furthermore, we verified that miR-3666 directly targeted IGF-1 by luciferase reporter assay. By using miR-3666 mimics, cell proliferation, migration, and invasion were suppressed, while being enhanced by the reduction of miR-3666. Knockout of IGF1 reverses the effect of the miR-3666 inhibitor on the malignant behavior of LECs. These results indicate the role of miR-3666/IGF-1 in LEC-EMT that offers new strategies for the therapy and prevention of PCO.

## 1. Introduction

Cataracts are the major cause of blindness in China, and it is also the main cause of blindness in most countries over the world [1, 2]. At present, surgery is the only effective treatment [3]. The PCO or posterior cataract is a common complication after cataract surgery, and it is also the main cause of postoperative visual acuity decline [4]. Studies have reported that the residual LECs generated by EMT play a critical role in the development of PCO [5].

EMT refers to the biological process in which epithelial cells are transformed into cells with interstitial phenotype through some specific procedures. It plays a vital role in embryonic development, a variety of fibrotic diseases, and cancer metastasis [6, 7]. PCO is one of the main reasons that affect visual quality after cataract surgery. The principle of formation is mainly caused by the surgical incision caused by cataract surgery, which leads to the release of various inflammatory factors in aqueous humor, stimulating the residual lens epithelial cells under the capsule [8, 9]. Subsequently, LECs undergo a series of biological behaviors, such as proliferation, migration, and transformation, which eventually lead to the opacity of the posterior capsule [10, 11]. Therefore, it is of great significance to explore the mechanism of EMT in LECs for cataract treatment.

IGF-1 has been reported to be involved in many diseases and promotes EMT in tumor cells [12, 13]. Moreover, IGF-1 has been reported to be related to the pathogenesis of diabetic ophthalmopathy. The level of IGF-1 in the vitreous of patients with diabetic retinopathy is increased [14, 15]. IGF-1 overexpression in transgenic mice results in neovascular glaucoma [16], and IGF-1 has been found to affect the protein composition of LECs, leading to cataracts [17]. However, the effect of IGF-1 on lens epithelial cell EMT is not clear.

The miRNAs are a kind of noncoding small RNAs that cause gene degradation or translation inhibition by binding to the complementary sequence of the target mRNA 3'-untranslated region. Accumulating evidence shows that miRNAs play an important role in PCO, such as miR-30a [18], miR-204-5p [19], miR-34a [20], and miR-486-5p [21]. The function of miR-3666 in the pathophysiological process of different types of cancer has been widely studied [22–24]. However, the function of miR-3666 in the pathogenesis of EMT in LECs has not been verified. In the present study, we found that the high expression of IGF-1 promotes the EMT process of HLECs, and miR-3666 bound to IGF-1 attenuated TGF-*β*2-induced EMT in HLECs.

## 2. Materials and Methods

### 2.1. Capsular Injury Model in Rats

1-month-old Wistar rats were purchased from Shanghai Laboratory Animal Co., Ltd (SLAC) (Shanghai, China). Animal care and experimental protocols complied with the guidelines of the Animal Ethics Committee of Harbin Medical University (number: sydwgzr2020-11). The rats had free access to water and food and were kept in normalized laboratory surroundings (12 h illumination/12 h dim cycle with lights on at 07 : 30 am, relative humidity: 45 ± 10%, temperature:20 ± 2°C). After anesthetized generally with pentobarbital sodium (Merck KGaA, Darmstadt, Germany) (70 mg/kg) and topically with Dicaine eye drops, a 1 mm incision was made at the transparent cornea at noon and filled with hyaluronic acid to maintain the state of the anterior chamber. After cutting off the anterior capsule, BSS solution was injected into the capsule to completely separate the lens cortex from the capsule. Then, the corneal incision was sutured. The occurrence of PCO was observed using a slit-lamp microscope at 0, 3, 7, 14, 21, and 28 days after operation [25]. All the animals were intraperitoneally injected with 3% pentobarbital sodium and were euthanized by excessive anesthesia with a dose of 90 mL/kg. Then, the eyes were enucleated and the posterior capsular tissue of the lens was removed for the experiments.

### 2.2. Cell Culture

Human lens epithelial cells SRA10/04 were purchased from ATCC (Manassas, VA, USA). The cells were cultured with a complete medium including 89% DMEM and 10% FBS (Biological Industries, Beit HaEmek, Israel) and kept in an incubator at 37°C and 5% CO_2_ saturated humidity.

The final concentration of TGF-*β*2 (PeproTech, Rocky Hill, NJ, USA) was 10 ng/ml. Before being collected for further analysis, the cells were cultured in the medium containing TGF-*β*2 for 48 hours.

### 2.3. Western Blot

Cells were lysed with RIPA buffer (CST, Danvers, MA, USA), and 45 ug proteins were run on an 8% SDS-polyacrylamide gel and then transferred onto the PVDF membrane. After 1 hour of blocking with 5% skim milk, the membranes were incubated with primary antibodies overnight at 4°C. The corresponding secondary antibodies were incubated at room temperature for 1 hour the next day. Primary antibodies against IGF-1 (DF6096, 1 : 500), vimentin (AF7013, 1 : 2000), E-cadherin (AF0131, 1 : 500), and *β*-actin (AF7018, 1 : 2000) were purchased from Affinity Biosciences (Jiangsu, China), with *β*-actin as an internal control. Subsequently, we washed the membranes (three times for 15 min, each wash) with TBST and incubated them with a goat antirabbit (1 : 3000, Abcam, Cambridge, MA, USA) or antimouse secondary antibody (1 : 3000, Abcam) for 2 h at 26 ± 2°C. An Odyssey infrared imaging system (Odyssey CLx, Biosciences, USA) was used to detect immunoreactivity.

### 2.4. qRT-PCR

The Trizol reagent was used to extract RNA from cells or tissues. NanoDrop 8000 (Thermo Scientific, Waltham, MA, USA) was used to detect the concentration and purity of RNA. The single-stranded cDNAs were synthesized from 1 *μ*g of RNA. The expressions of mRNAs and miRNAs were quantified by RT-PCR with SYBR Green I (Thermo Fisher Scientific, Inc). The primer sequences of human genes are shown in Table 1.

### 2.5. miRNA and Plasmid Transfection

The LECs were plated until the cell density reached 80% confluency of dishes to transfect. The miRNAs/inhibitors/plasmids were transfected with Lipofectamine 2000 (Invitrogen, Carlsbad, CA). miR-3666 mimics/inhibitors were bought from RiboBio (Guangzhou, China) and plasmid of IGF-1 or short hairpin RNA of IGF-1 (sh-IGF-1) were constructed by GeneChem (Shanghai, China).

### 2.6. EdU Assay

EdU cell proliferation kit (RiboBio, Guangzhou, China) was used to test proliferation. LECs were seeded in 24-well plates. After miRNA or plasmid transfection for 48 h, cells were maintained with 200 uL 50 uM EdU for 2 h. Apollo dye solution (red) was used to stain the proliferating cells, and nucleic acids were stained with DAPI (blue) according to the protocols [26] and then photographed.

### 2.7. Wound-Healing Assay

To test the cell migration ability of LECs, a wound-healing assay was performed. LECs were plated and cultured with FBS-free medium in 6-well plates until the cells formed a confluent monolayer and then were scratched using a 100 *μ*L pipette tip. The scratch wounds were captured using microscopy at 0 and 24 h. The wound area was analyzed by Image J.

### 2.8. Luciferase Reporter Assays

To verify if IGF-1 was a target of miR-3666, the 3'-UTR of IGF-1 including the predicted binding sites wild (wt) or mutated (Mut) binding sites were inserted into the pmirGLO vector. The reporter plasmids of IGF-1 were cotransfected with miR-3666 mimics or miR-NC. Luciferase activities were measured by using a dual-luciferase reporter assay kit (Promega, Madison, Wisconsin, USA) after 24 h.

### 2.9. Matrigel Transwell Assay

24-well Matrigel transwell assay (Corning, San Diego, CA, USA) was used to investigate cell invasion. 2 × 10^5^ LECs were seeded on the cell culture insert precoated with 1 *μ*g/*μ*L Matrigel (BD Biosciences). A medium with FBS was used to stimulate invasion in the bottom of the wells. After 48 h, the invasion cells were stained with a 0.1% crystal violet solution. The number of invading cells was counted under the microscope.

### 2.10. Statistical Analysis

Data are shown as mean ± SEM. The unpaired Student's *t*-test or one-way ANOVA was used to compare the groups. *P* < 0.05 was considered significant.

## 3. Results

### 3.1. IGF-1 Was Upregulated in OPC and TGF-*β*2-Induced HLEC-EMT

We constructed an injury-induced OPC model in rats. QRT-PCR confirmed that the level of IGF-1 was upregulated in the lens posterior capsule tissue of the OPC model compared to the control, as shown in Figure 1(a). We then tested the IGF-1 expression in TGF-*β*2-induced HLEC-EMT. We verified that the TGF-*β*2 exposure promoted the IGF-1 mRNA level at 48 h, as shown in Figure 1(b). The result of the western blot revealed that IGF-1 protein was increased after treatment with TGF-*β*2, as shown in Figures 1(c) and 1(d).

### 3.2. Overexpression of IGF-1 Promotes the EMT of HLECs

To analyze the potential effects of IGF-1 in the EMT of LECs, we constructed an IGF-1 plasmid and confirmed the overexpression efficiency using qRT-PCR, as shown in Figure 2(a). After being transfected with the IGF-1 plasmid, the epithelial cells marker CDH1 mRNA level was decreased, as shown in Figure 2(b), and the mesenchymal-related marker vimentin mRNA level was increased, as shown in Figure 2(c). Overexpression of IGF-1 also downregulated the protein level of E-cadherin and upregulated the vimentin protein level, as shown in Figures 2(d) and 2(e), respectively. Subsequently, an in *vitro* wound-healing assay demonstrated that IGF-1 overexpression promoted the ability of HLECs to close a wound, indicating that IGF-1 promotes a cell migratory phenotype, as shown in Figures 2(f) and 2(g). Furthermore, Matrigel invasion experiments displayed that upregulated IGF-1 promoted cell invasion, as shown in Figures 2(h) and 2(i). EdU staining was conducted to detect cell proliferation activity, and we found that IGF-1 enhanced the proliferation ability of HLECs, as shown in Figures 2(j) and 2(k). Collectively, the abovementioned results show that forced expression of IGF-1 promotes the EMT phenotype of HLECs.

### 3.3. Silencing IGF-1 Alleviated TGF-*β*2-Induced EMT of HLECs

Since the overexpression of IGF-1 has suggested a role in promoting EMT, we next validated whether silencing IGF-1 has an anti-EMT effect on HLECs. We constructed an IGF-1 short hairpin RNA (sh-IGF-1) and performed the functional assays, as shown in Figure 3(a). The expressions of E-cadherin and vimentin were tested by qRT-PCR and western blot. After IGF-1 silencing, we found that E-cadherin levels were increased, as shown in Figures 3(b)–3(e), whereas levels of vimentin were decreased in TGF-*β*2-induced HLECs-EMT, as shown in Figures 3(c)–3(e). The wound-healing assay showed sh-IGF-1 decreased cell motility induced by TGF-*β*2, as shown in Figures 3(f) and 3(g). Strikingly, sh-IGF-1 inhibited HLEC invasion and migration induced by TGF-*β*2, as shown in Figures 3(h)–3(k).

### 3.4. IGF-1 Was a Potential Target of miR-3666

It has been reported that microRNAs regulate the gene's expression and function. To clarify the regulatory relationship between miRNAs and IGF-1, we used the miRNA target identification tool TargetScan 7.2 (http://www.targetscan.org/vert_72/) to search for potential microRNAs binding with IGF-1. We identified miR-3666 which contained potential-binding sites on 3'-UTR of IGF-1, as shown in Figure 4(a). Luciferase reporter vectors were constructed with the 3'-UTR sequence of IGF-1 containing the putative binding site for miR-3666. The luciferase activity was suppressed with wild-type IGF-1 (IGF-1-wt) but not with the mutated IGF-1 vector (IGF-1-mut), as shown in Figure 4(b). Contrary to IGF-1, low miR-3666 expression was observed in cataract tissues, as shown in Figure 4(c), and HLECs treated with TGF-*β*2, as shown in Figure 4(d). Overexpression of miR-3666 with mimics suppressed the expression of IGF-1, which further proved the regulatory relationship between them, as shown in Figure 4(e).

### 3.5. Enhanced Expression of miR-3666 Attenuates EMT of LECs

To further validate the role of miR-3666, HLECs were transfected with miR-3666 mimics and miR-NC with or without TGF-*β*2, respectively. The mRNA level of CDH1 was high expression and vimentin was downregulated when treated with miR-3666 mimics in TGF-*β*2-induced cells, as shown in Figures 5(a) and 5(b), respectively. The protein levels that E-cadherin was upregulated and vimentin was downregulated in the miR-3666 mimics group were further detected by western blot, as shown in Figures 5(c) and 5(d). Wound healing and invasion assays demonstrated that the migratory capacity and invasion ability of HLECs were markedly inhibited by miR-3666 mimics, as shown in Figures 5(e)–5(h). EdU assay indicated that proliferating cells were decreased with the presence of miR-3666 mimics, as shown in Figures 5(i) and 5(j). As has been reported in human tumors, miR-3666 impeded the EMT process of HLECs.

### 3.6. Inhibition of miR-3666 Promotes EMT by Regulating IGF-1

We further explored the effect of the miR-3666 inhibitor and the biological regulatory relationship between miR-3666 and IGF-1 in *vitro*. We constructed the miR-3666 inhibitor and the negative control inhibitor and verified their functions, as shown in Figure 6(a). According to the results of qRT-PCR and western blot, we found that upon being treated with the miR-3666 inhibitor, E-cadherin levels were decreased, as shown in Figures 6(c)–6(f), whereas the levels of IGF-1 and vimentin were increased, as shown in Figures 6(b)–6(f), in TGF-*β*2-induced HLEC-EMT. By transfecting sh-IGF-1 into HLECs, we found that silencing IGF-1 partially reversed the EMT promoting function of the miR-3666 inhibitor. As expected, the miR-3666 inhibitor promoted the migration, invasion, and proliferation of HLECs, but the silencing of IGF-1 partially restored cell function, as shown in Figures 6(g)–6(l).

## 4. Discussion

This study shows that IGF-1 is directly related to the EMT process of HLECs. Overexpression of IGF-1 promoted the proliferation, migration, invasion, and EMT of HLECs, whereas knockout of IGF-1 significantly inhibited the EMT phenotype induced by TGF-*β*2.

Previous studies have shown that IGF-1 receptors are widely distributed in the eyes [27]. For example, there were IGF-1 receptors in lens epithelial cells, so IGF-1 is capable of stimulating lens cell differentiation by binding its receptors [28], which is one of the reasons leading to PCO. Crystallin aggregation is also the cause of cataracts; it is described that IGF1-1 affects the total ratio of *β* and *γ* crystallin to *α* crystallin in lens fiber cells, which may make the lens susceptible to cataracts. In humans, mutations of IGF-1 can reduce retinal angiogenesis [29]. It is suggested that IGF-1 may play a critical role in the occurrence and development of ocular complications. Our study clearly defines the effect of IGF-1 on LECs.

In addition, we used a bioinformatics website to screen valuable microRNAs which bind to IGF-1 to regulate lens epithelial cell proliferation and predicted that miR-3666 may regulate IGF-1 by binding to the 3' UTR of IGF-1. The luciferase reporter gene experiment verified the targeting relationship between them. Overexpression of miR-3666 can inhibit the proliferation, migration, invasion, and interstitial phenotype of HLECs, whereas knockout of IGF-1 reverses the effect of the miR-3666 inhibitor on the malignant behavior of HLECs [30]. These results highlight the role of miR-3666/IGF-1 in lens EMT and provide a new strategy for the prevention and therapeutic method of PCO.

At present, most of the studies of EMT in PCO are focused on cell and animal experiments, and the mechanism is complex and needs to be further explored. Understanding the specific molecular mechanism of the occurrence and development of LEC-EMT is very important for the treatment of PCO and also provides ideas for the prevention of PCO from a new point of view.

## 5. Conclusion

In summary, the present study provides evidence for the miR-3666/IGF-1 pathway involved in TGF-*β*2-induced HLEC-EMT. miR-3666 acts as an endogenous sponge of IGF-1 and regulates EMT phenotype and cell activity. These findings provide a novel insight into understanding that the mechanisms of HLEC-EMT provide in vitro support for the specific pathogenesis of PCO. Our results indicate the potential therapeutic target to heal the damaging process after cataract surgery.

## Figures and Tables

**Figure 1:** The expression of IGF-1 in PCO and TGF-*β*2 induced HLECs. (a) The mRNA expression of IGF-1 in the posterior capsule tissue of the PCO model and healthy control was detected by qRT-PCR, *n* = 6. (b) The expression level of IGF-1 mRNA in TGF-*β*2 induced HLECs was determined by qRT-PCR, *n* = 6. (c) The protein level of IGF-1 was confirmed in TGF-*β*2-induced HLECs and the control group by western blot. (d) Statistical data of western blot, *n* =  4. ^*∗*^*p* < 0.05; ^*∗∗*^*p* < 0.01.

**Figure 2:** Overexpression of IGF-1 results in EMT in HLECs. (a–c) qRT-PCR was used to confirm mRNA expression of IGF-1, CDH1, and vimentin to detect the effect of IGF-1 overexpression in HLECs, *n* = 6. (d) The protein levels of IGF-1, E-cadherin, and vimentin were determined by western blot to detect the effect of IGF-1 overexpression in HLECs. (e) Analysis of western blot, *n* = 4. (f) The wound-healing assay revealed that overexpression of IGF-1 increased cell migration in HLECs. (g) Analysis of wound-healing assay, *n* = 6. (h) Transwell assay showed the invasion ability of HLECs was promoted by IGF-1. (i) Analysis of Transwell assay, *n* = 6. (j) EdU staining illustrated that forced expression of IGF-1 promoted cell proliferation. (k) Analysis of EdU staining, *n* = 6. ^*∗*^*p* < 0.05; ^*∗∗*^*p* < 0.01.

**Figure 3:** Inhibition of IGF-1 ameliorated HLEC-EMT after TGF-*β*2 was treated. (a) qRT-PCR was used to verify the efficiency of sh-IGF-1, *n* = 6. (b, c) Silencing IGF-1 reversed TGF-*β*2-induced mRNA expression of CDH1 and vimentin, which was measured by qRT-PCR assay. (d) Using western blot to investigate the effect of sh-IGF-1 with or without TGF-*β*2 on the level of IGF-1, E-cadherin, and vimentin proteins. (e) Analysis of western blot, *n* = 4. (f) Wound healing revealed that inhibiting IGF-1 ablated the cell migration induced by TGF-*β*2. (g) Analysis of wound healing assay, *n* = 6. (h) Transwell assay showed that invasion ability of HLECs was inhibited by sh-IGF-1. (i) Analysis of Transwell assay, *n* = 6. (j) EdU staining revealed that knockdown of IGF-1 inhibited cell proliferation induced by TGF-*β*2. (k) Analysis of EdU staining, *n* = 6. ^*∗*^*p* < 0.05; ^*∗∗*^*p* < 0.01.

**Figure 4:** Identification of miR-3666 as a master miRNA regulating the IGF-1. (a) Predicted binding sites of IGF-1 and miR-3666. IGF-1-Mut, mutated binding site. (b) Luciferase activities of chimeric vectors with IGF-1 containing wild-type or mutated. (c) The expression of miR-3666 in posterior capsule tissue of the PCO model and healthy control was detected by qRT-PCR, *n* = 6. (d) The expression of miR-3666 in HLECs with or without TGF-*β*2 was determined by qRT-PCR, n = 6. (e) The effect of miR-3666 on IGF-1 mRNA expression, *n* = 6. ^*∗*^*p* < 0.05; ^*∗∗*^*p* < 0.01; NS, not significant.

**Figure 5:** Overexpression of miR-3666 attenuated TGF-*β*2-induced EMT in HLECs. (a, b) miR-3666 mimics reversed TGF-*β*2-induced mRNA expression of CDH1 and vimentin, which was measured by qRT-PCR. (d) Using western blot to investigate the effect of miR-3666 mimics with or without TGF-*β*2 on the level of IGF-1, E-cadherin, and vimentin proteins. (e) Analysis of western blot, *n* = 4. (f) Wound healing revealed that miR-3666 mimics ablated the increased cell migration induced by TGF-*β*2. (g) Analysis of wound-healing assay, *n* = 6. (h) Transwell assay showed that the invasion ability of HLECs was inhibited by miR-3666 mimics. (i) Analysis of Transwell assay, *n* = 6. (j) EdU staining illustrated that miR-3666 mimics inhibited cell proliferation induced by TGF-*β*2.

**Figure 6:** IGF-1 was necessary for promoting the EMT effects of the miR-3666 inhibitor. (a) qRT-PCR was used to detect the silencing efficiency of the miR-3666 inhibitor. *n* = 6. (b–d) Silencing IGF-1 reversed miR-3666 inhibitor-induced mRNA expression of IGF-1, CDH1, and vimentin, which was measured by qRT-PCR. *n* = 6. (e) Using western blot to investigate the effect of sh-IGF-1 with or without the miR-3666 inhibitor on the level of IGF-1, E-cadherin, and vimentin protein. (f) Analysis of western blot, *n* = 4. (g) Wound-healing tests showed that inhibition of IGF-1 ablated the cell migration induced by the miR-3666 inhibitor. (h) Analysis of wound-healing assay, *n* = 6. (i) Transwell assay showed that the miR-3666 inhibitor-induced invasion ability of HLECs was inhibited by sh-IGF-1. (j) Analysis of Transwell assay, n = 6. (k) EdU staining showed that silencing of IGF-1 inhibited cell proliferation induced by the miR-3666 inhibitor. (l) Analysis of EdU staining, *n* = 6. ^*∗*^*p* < 0.05; ^*∗∗*^*p* < 0.01.

**Table 1:** The sequences (human or rats) of the required primers.

Name	Forward primer (5'–3')	Reverse primer (5'–3')
GAPDH	ACCACAGTCCATGCCATCAC	TCCACCACCCT GTTGCTGTA
miR-3666	ACGAGACGACGACAGAC	CAGTGCAAGTGTAGATGCCGA
U6	GCUUCGGCAGCACAUAUACUAAAAU	CGCUUCACGAAUUUGCGUGUCAU
IGF-1	CAGCAGTCTTCCAACCCAAT	GCTGACTTGGCAGGCTTGAG
CDH1	CTGAGAACGAGGCTAACG	CCACCATCATCATTCAATATG
N-cadherin	ACACTGGTGGCACTACTAAG	TACACAATACAGAGGCAAAG
IGF-1(rats)	CTTTACCAGCTCGGCCACA	TTGGTCCACACACGAACTGAAG

## Data Availability

The simulation experiment data used to support the findings of this study are available from the corresponding author upon request.
